# Innovation in Brain Tumor Treatment: A Nurse Perspective

**DOI:** 10.7759/cureus.20037

**Published:** 2021-11-30

**Authors:** Alexandria K Reddelle

**Affiliations:** 1 Community Care, Department of Veterans Affairs Medical Center, Columbus, USA

**Keywords:** surgical intervention, implementation, cancer, treatment, gammatile, brain tumor

## Abstract

GammaTile is a newer development in brain tumor treatment providing surgically targeted treatment for patients suffering from both primary and recurrent tumors. This article addresses the implementation of this new treatment. The article provides an overview of brain tumors, their diagnosis, and more traditional, widely used treatments. The article discusses implementing a new treatment and the processes involved. It discusses the first patient case for the Columbus, OH area and makes recommendations for future uses of this innovative treatment in other areas of the body.

## Introduction

Brain tumors significantly impact the lives of patients and families. According to the National Brain Tumor Society (NTBS) [1], there are approximately 700,000 Americans diagnosed with a primary brain tumor, while 63% are considered benign, 37% are found to be malignant. Data collected show that males have a higher instance of occurrence, accounting for approximately 58%, according to the National Brain Tumor Society [1].

In the year 2020, brain tumors were the 10^th^ leading cause of death [1], accounting for approximately 18,020 adults, with 10,190 being men and 7,830 being women. The estimated five-year survival rate is approximately 36% under age 40, over age 40 is approximately 21% survival rate [2]. In 2021, an estimated 84,170 patients will receive a brain tumor diagnosis [1].

Brain tumors are separated into two distinct categories, primary and metastatic; primary tumors arise directly from the tissues of the brain, while metastatic tumors are caused by cancer cells spreading (metastasizing) to the brain from a different part of the body. Glioblastoma (GBM) is the most commonly diagnosed primary brain tumor, comprising 14.5% of all brain tumors. GBMs account for 48.6% of malignant tumors [1].

Treatments can vary, and there are no guarantees. Treatment is dependent on tumor size, the type of tumor present, the grade of the tumor, location in the brain (with focus on vital portions tumor affects), metastasis in the CNS or the body, the side effects that may occur, and the overall health of the individual patient [2].

Surgery, chemotherapy, and external beam radiation (EBT) are the most widely used treatment for these tumors. Additional treatment options include Gamma knife radiosurgery and Neuroblate (Laser interstitial thermal therapy) and Optune (tumor treatment fields) [3].

Despite the advancements in treatment for brain tumors, they remain a significant underserved medical problem affecting the lives of thousands. Not only are the patients affected, but the families suffer as well. A continual search to find the cure for this treacherous disease is ongoing. Current treatments not only aim to cure these tumors but to advance the lives of the patients. Diagnosis can be precarious; however, their identification has been standardized, making diagnosis more accurate and efficient. This allows for appropriate diagnosis and treatment options [4]. 

## Case presentation

Brain tumor grading system

CNS tumors are graded by a preset scale. The WHO has set forth a CNS tumor classification system. Classification is organized based on the origin cell, even though there has been a significant move to use molecular markers [4,5]. The criteria for classification are included in Table 1.

Criteria for classification

**Table 1:** Criteria for Brain Tumor Classification [1]

Grade Description	WHO Grade	Characteristics	Types
Low Grade	I	Benign possibly, curable w surgery slow growing High survival rate	Pilocytic astrocytoma Craniopharyngioma Gangliocytoma Ganglioglioma and Meningioma
Low Grade	II	Slow growing, some infiltration may recur at higher grades	Diffuse astrocytoma Pineocytoma Pure Oligodendrogolioma
High Grade	III	Malignant infiltrative recur at higher grade	Anaplastic astrocytoma Anaplastic ependyoma Anaplastic oligodendroglioma
High Grade	IV	Malignant aggressive, rapid growth severely infiltrative rapid recurrence prone to necrosis	Glioblastoma (GBM) Pineoblastoma Medulloblastoma Ependymoblastoma (aana, 2020)

The World Health Organization (WHO) has identified tumor types and classified them based on their primary characteristics. This enables quick identification and treatment options (Table 2).

Tumor classification

**Table 2:** Tumor Classification [6]

Grade	Classification
I	Slow growing non-malignant high survival rate
II	Meet one criterion on list slow growing High recurrence rate both malignant and non-malignant
III	Meet two criteria malignant high recurrence rate
IV	Meets 3-4 criteria rapidly reproduce extremely aggressive malignant

GammaTile treatment

GammaTile (GT) is a more recently developed treatment for brain tumors that have shown significant results. Developed by a team that was comprised of neurosurgeons, radiation oncologists, and radiation physicists. This innovative treatment provides immediate treatment approved for use in all cranial tumors, both recurrent and primary. 

Because GT is placed at the time of surgical resection, radiation to any residual tumor begins immediately, and compliance with the treatment plan is assured. Because of its targeted placement and immediate compliance with treatment, GT has been shown to significantly increase the survival rate and improve the quality of life. Based on the results of precommercial studies, GT increased the survival rates significantly over both one-year and two-year periods by approximately 30% [7].

Recurrent GBM Median Survival Rates [7] GT studies have shown through the use of GT as an alternative therapy, the survival rate among patients with recurrent brain tumors achieved a median of 16.7 months as compared to patients treated with traditional or no treatment, in whom the survival rate was only 9.7 months.  

Brain metastases patient recurrence-free at one year: studies also showed the rate of non-recurrence after one year 83% of patients treated with GT were tumor-free, while only 33% of traditionally treated patients had no recurrence [7].

Brain metastases patient recurrence-free at two years: after two years, the rate of being free from tumor recurrence was 89%. Of patients who received traditional or no treatment, the progression-free rate at two years was only 52%. The use of GT as a treatment option significantly increased the likelihood that the patient would not have a recurrence [7]. The recurrence-free statistics are discussed in Table 3.

**Table 3:** Recurrence-Free Statistics [7]

Recurrence free survival rates	Patients who received GT treatment	Patients who chose traditional or no treatment
Overall survival	16.7 months	9.7 months
No brain metastases at one year	83%	33%
No brain metastases at two years	89%	52%

Our first patient treated with GT was a 62-year-old female named ZL. Diagnosed with colon and rectal cancer in August 2019, ZL underwent a multitude of traditional treatments. These treatments involved chemotherapy and external beam radiation (EBR). Despite the aggressive treatment, ZL's condition worsened. ZL developed metastasis in her brain due to metastasis. In Feb 2020, ZL underwent a craniotomy for tumor resection. Over the next few months, the tumor regrew in her brain. ZL was a perfect candidate for GT. We worked closely with the GT team to calculate the approximate number of tiles needed and to coordinate timely delivery. We received the appropriate number of tiles in the facility on June 26, 2020. The tiles were delivered directly to the nuclear-med lab, and the physicist was on-site to verify the contents for accuracy. Due to the timing of the order delivery and the half-life of Cs-131, as compared to the time of surgery, the tiles were made more radioactive than typically. This process was used to accommodate for the delay in delivery to surgery to ensure the correct radioactive strength was present when placed. On June 29, 2020, ZL underwent a second craniotomy for tumor resection. During the operative procedure, specimens were taken to the lab for stat processing to confirm tumor cells. Once tumor presence was confirmed, the team was called to the operating suite. After completing the resection of the tumor, the radiation oncologist passed each tile individually to the surgeon. The tiles were placed in a blanket configuration covering the tumor bed. This took approximately two minutes to complete. The cranium was then closed, and ZL was taken directly to the ICU for recovery. The following day, ZL received a standard repeat scan, which showed tiles remained in place. ZL did return to surgery a few days later for cerebrospinal fluid (CSF) leak repair, which was deemed unrelated to the GT placement by the surgeon. ZL returned to her home the following week, and her recovery went well, as expected. This new treatment proved to be successful for ZL. In August 2020, ZL spoke about her experience through a video [8].

Because of the advanced technology through GT, she was able to return to her active lifestyle and live a fuller life than she would have under traditional conditions.

## Discussion

While traditional treatments have shown success, they are not without their drawbacks. The development of new technologies and alternatives to combat such a deadly diagnosis is imperative to prolonging life more positively. Traditional radiation therapy cannot preserve surrounding brain tissue and can leave a large section of necrotic areas that can impair a person's ability to function normally. As compared to traditional treatment, GT placement being strategically placed allows for a more targeted treatment decreasing the areas of necrosis around the tumor site. [3,7]. Other treatments discussed, including but not limited to chemotherapy and EBT, require an extensive physical component for treatment, unlike GT, which has an immediate response and full compliance with minimal to no side effects [1,2,4]. Using traditional treatment post tumor removal also necessitates a waiting period of six weeks for the incision to heal before any treatments. Through the targeted and strategically intraoperative placement, GT allows the patients to receive treatment immediately, therefore minimizing the risk of recurrence. 

Being a newer treatment, GT was only available at a select few hospitals. Implementing this treatment option took multiple steps. The first step was to complete the research, determine what type of opportunity this program presented for the facility, and the population it served, along with essential personnel needed for this team were then identified. Next, a process map was developed. This map covered the identification of the patient as a candidate by the neurosurgeon to the placement of GT and recovery. The next step was to present a prospectus for financial considerations, which was necessary to be done for each patient, as insurance reimbursement differs by the plan. The implementation program occurred over several months; however, it could feasibly be accomplished in a matter of weeks, dependent upon the facility. Once the preliminary tasks were completed, an organizational meeting was held. Individual tasks were assigned, and regular progress meetings were scheduled. The key players in implementing this program were not only the surgeon but recruiting a radiation oncologist was essential to the success of the program. Other team members included the clinical manager of neurosurgery, the director of surgical services, radiation safety officer (RSO), physicist, nuclear-med lab manager, finance, staff involved, and the marketing team. Once the program was instituted, the process map was utilized to ensure the individual steps were followed, and all aspects of the procedure were accomplished timely. 

## Conclusions

GT was developed to extend the lives of patients suffering from recurrent brain tumors. GT has now been approved by the FDA for all cranial neoplasms regardless of recurrent or primary. This treatment has extended the lives of many individuals who would not be here today if they had not received treatment with GT. GT offers patients immediate treatment that is targeted at the exact location needed. There is no need to wait weeks for the incision to heal after surgery, and there is no need to endure multiple trips to the clinics and outpatient treatment centers. This not only helps the patient return to normal life more quickly but also decreases the burden on the families involved. Instituting this program, while met with some obstacles, proved to be beneficial for the patient, and I believe it will be beneficial for future patients. Patients want close-to-home care, and they want the care to be innovative, comprehensive, and minimally invasive in their daily lives. The next step is to transition this treatment for use in other malignant tumors. Obtaining approval to use in spinal tumors would be the next step as GT could show similar long-term results. Expanding this treatment to incorporate its use with other cancers such as uterine, renal, and breast could prove beneficial as well. While the current statistics look promising, further evaluation and research are necessary before its widespread usage.
